# MR Image Classification for Brain Tumor Texture Based on Pseudo-Label Learning and Optimized Feature Extraction

**DOI:** 10.1155/2022/7746991

**Published:** 2022-04-04

**Authors:** Qianqian Xu, Huachang Xu, Jie Liu, Mingxia Zhou, Min Li, Jinhui Xu, Hong Zhu

**Affiliations:** ^1^School of Medical Information and Engineering, Xuzhou Medical University, Xuzhou, China; ^2^Department of Computer Science and Engineering, State University of New York at Buffalo, Buffalo, USA

## Abstract

Brain tumors are the deadliest and most difficult to treat of all forms of cancer. Preoperative classification of brain tumors is conducive to the development of corresponding treatment plan. Take pituitary tumors as an example. Precisely judging the image data of pituitary tumor texture before surgery can provide a basis for the selection of surgical plan and prognosis. However, the existing methods require manual intervention, and the efficiency and accuracy are not high. In this paper, we proposed an automatic brain tumor texture diagnosis method for uneven sequence image data. First, for the small sample of pituitary tumor MRI image data, the T1 and T2 sequence data are uneven or missing; we used the CycleGAN model to perform data conversion between different domains to obtain a completely sampled MRI spatial sequence. Then, we used texture analysis+pseudo-label learning to label pituitary tumor data of some unknown labels. After that, we used the improved U-Net model based on CBAM to optimize feature extraction for pituitary tumor image data. Finally, we used the CRNN model to classify the degree of pituitary tumor texture based on the advantages of sequence data. The entire process only needs to provide labels for the entire sequence data, and the efficiency is greatly improved, with an accuracy rate of 94.23%.

## 1. Introduction

Brain tumors, including various intracranial tumors, are classified into benign and malignant. In recent years, the incidence of intracranial tumors has been on the rise. According to statistics, intracranial tumors account for about 5% of systemic tumors and 70% of childhood tumors. Due to its swelling and infiltrating growth, once occupying a certain space in the skull, whether it is benign or malignant in nature, it will inevitably increase intracranial pressure, compress the brain tissue, cause central nervous system damage, and endanger the lives of patients. Take pituitary tumors as an example. A pituitary tumor is one of the most common intracranial tumors. The pituitary tumor has a serious disease burden, and its treatment involves neurosurgery, biological therapy, and radiation therapy [1]. The softness and density of pituitary tumors are related to many key issues, such as whether surgery is required, what kind of surgery to use, and what is the expected surgical effect. However, due to the nature of cranial cavity, it is often difficult to determine the softness of pituitary tumors before surgery. Therefore, how to accurately determine the softness of pituitary tumors in a noninvasive manner has become an important issue [2]. With the advancement of medical imaging technology, Magnetic Resonance Imaging (MRI), Computed Tomography (CT), and other imaging methods have become an important basis for assisting doctors in diagnosis. Therefore, it is very valuable to dig out deep quantitative information (such as the softness of pituitary tumors) that clinicians cannot detect with the naked eye from medical images.

With the popularity of artificial intelligence, deep learning is increasingly used in medical image processing. B. Zhou and S.K. Zhou [3] proposed a dual-domain recurrent network for rapid MRI reconstruction. This kind of network can recover *k*-space and images at the same time and finally reconstruct high-quality MRI. Balakrishnan et al. [4] proposed the VoxelMorph framework for deformable pairwise medical image registration, which can speed up the analysis and processing of medical images. Hashimoto et al. [5] developed a new method of cancer subtype classification based on the Convolutional Neural Network (CNN) in combination with multi-instance, domain adversarial, and multiscale learning framework. An autoencoder is an unsupervised model in deep learning which can automatically extract many deep features from the medical image datasets. Gu et al. [6] proposed a context encoder network for 2D medical image segmentation. This network consists of a feature encoder module, a context extractor, and a feature decoder module, which can extract more advanced information and keep the space information. These results all suggest that the autoencoder has good utility and robustness in image feature extraction and model efficiency. Thus, it is quite suitable to use the autoencoder as a feature extractor in medical image processing.

These types of deep learning often require large amounts of labeled data. However, due to privacy concerns, medical image data used in practice are often small samples with incomplete labels. This motivates us to propose in this paper a semisupervised brain tumor image classification method based on CycleGAN, pseudo-label, and optimized feature extraction. Our rationale behind using CycleGAN is that medical images are often incomplete and often have data missing. CycleGAN enables us to generate additional data to make up the missed ones. Also, medical images are often unlabeled, which could make the classification task considerably more challenging. To resolve this issue, our idea is to use the method of texture analysis+pseudo-label learning to label them. Furthermore, we propose a new feature extractor based on improved U-Net and adopt some attention mechanism to extract brain tumor features and perform adaptive optimization. The feature extractor can effectively extract features from medical images. Finally, for sequence data, our method feeds the optimized feature sequences into a Convolutional Recurrent Neural Network- (CRNN-) based classifier to complete the classification of brain tumor texture. In this paper, we use MRI of the pituitary tumor as an example for experiments.

## 2. Methods

### 2.1. Theoretical Basis

#### 2.1.1. Pseudo-Label Learning

Pseudo-label learning is a semisupervised learning method. Pseudo-label learning refers to the use of existing labeled data to train a model, and then, use the model to predict and label unlabeled data. Pseudo-label learning generally includes three steps. First, use the labeled data to train a model, then use the model to make label predictions on the unlabeled data, and finally use the pseudo-labeled data and the labeled data to retrain the model.

#### 2.1.2. GRU

Gated recurrent unit (GRU) [7] is a kind of RNN, and its internal structure is similar to LSTM. GRU uses an update gate and reset gate. Compared with LSTM, it has one less gate, so it is easier to calculate. GRU is widely used because it can achieve the same functions as LSTM while reducing parameters.

#### 2.1.3. CBAM

The Convolutional Block Attention Module (CBAM) [8] is an attention mechanism module. It combines channels and space, so it has a better effect than the attention mechanism that only focuses on channels. The output result of convolutional layers with a CBAM structure will first pass through the channel attention module and then through the spatial attention module to get the final result. CBAM can make the model pay more attention to effective features, thereby improving the efficiency of feature extraction and thus the accuracy of the model.

### 2.2. Pituitary Tumor Sequence Data Amplification Using CycleGAN

MRI images of patients with pituitary tumors usually consist of different forms of spatial sequences, such as T1WI, T2WI, T1C, and T2FLAIR. The pituitary tumor dataset used in this paper is mainly composed of T1 and T2 spatial sequence images. In actual pituitary tumor MRI image acquisition, due to various practical reasons, such as data loss, data in a certain domain (such as T2) is usually missing. In order to supplement these missing data, we need to generate images of another domain based on the images of one domain and then merge them to generate a more complete dataset.

CycleGAN [9] can convert images of two domains into each other. CycleGAN includes two generators and two discriminators. In view of the characteristics of pituitary tumor data, we chose CycleGAN to complete the supplement of missing data. It can help us to complete the two-way conversion from the T1 domain to the T2 domain and from the T2 domain to the T1 domain. The network structures of the CycleGAN generator and discriminator used in this experiment are shown in Figures 1 and 2, respectively. The convolution layer of the generator consists of Conv2D, leaky ReLU, and instance normalization. The first three deconvolution layers consist of UpSampling2D, Conv2D, ReLU, and instance normalization, and the last deconvolution layer consists of UpSampling2D, Conv2D, and Tanh. The convolution layer of the discriminator consists of Conv2D, leaky ReLU, and instance normalization. Through the mutual conversion of the T1 domain and T2 domain, we expanded the number of slices in each domain to 12, making a total of 24 images of pituitary tumors for each patient to form a complete dataset.

### 2.3. Data Augmentation Method Based on Texture Analysis and Pseudo-Label Learning

There are 374 cases of pituitary tumor imaging data in this experiment, but only 137 cases have soft and flexible labels. In order to expand pituitary tumor data and improve the data utilization, we used a method of texture analysis+pseudo-label learning to label the remaining 237 unlabeled pituitary tumor data.

We first performed texture analysis on the labeled pituitary tumor images, such as extracting their texture or statistical features, to find the decisive parameters. Then, we used these analyzed parameters as reference standards to label unlabeled data. In order to improve the accuracy of the labeling, we extracted part of the data labeled by texture analysis and part of the data with real labels to synthesize a new labeled training set. Then, we used this new dataset to train a model; here, we chose the GRU model. Finally, we used the trained GRU model to predict the unlabeled data again, generate the final label, and complete the pseudo-label learning. The specific process is shown in Figure 3.

**Step 1 .**

Using texture analysis method to label the unlabeled pituitary tumor data.

**Step 2 .**

Randomly extracting 50% data from 237 cases of pseudo-label data.

**Step 3 .**

Randomly extracting 20% of the 137 cases with labeled data as the test set and synthesizing the new training set with remaining data and 119 cases of pseudo-label data.

**Step 4 .**

Using the GRU model to train the new training set.

**Step 5 .**

Using the trained model to predict 237 cases of unlabeled data to obtain the final data labels.

### 2.4. Classifying Pituitary Tumor Texture Based on Adaptively Optimized Texture Extraction

We divided the classification model of pituitary tumor images into two parts: feature extraction and final classification. For the feature extraction of pituitary tumors, we adopted a feature extractor based on improved U-Net and added CBAM between the encoder and the decoder. For the final classification, we used a CRNN-based classifier.

#### 2.4.1. Adaptive Optimization of Feature Extraction

For the feature extractor, an encoder composed of dense blocks, a 1∗1 convolutional layer, and a 2∗2 AvgPooling layer is used to extract the features of pituitary tumor MRI sequence data. Each dense block consists of 4 convolutional layers with 64, 64, 128, and 128 kernels, respectively. The kernel size of each convolution layer is 1∗1, 3∗3, 3∗3, and 1∗1. Each convolutional layer uses leaky ReLU as the activation function. Dense blocks can enhance the feature propagation ability of pituitary tumor images due to dense connections, while convolutional layers and pooling layers are used to reduce the dimensionality. The entire encoder uses two such dense blocks.

The decoder consists of residual blocks, an upsampling layer, and a convolutional layer and is used to generate a spatial sequence with the same spatial dimensions as the original image. Each residual block consists of 4 convolutional layers with 64, 64, 128, and 128 kernels, respectively. The kernel size of each convolution layer is 1∗1, 3∗3, 3∗3, and 1∗1. Each convolutional layer uses leaky ReLU as the activation function. The residual block is used to compress the dimensionality of the feature map, and the upsampling layer and convolutional layer are used to perform the dimensionality upgrade operation. The use of residual structure can help us increase the depth of the network while avoiding the disappearance of gradients, thereby improving the effect of MRI spatial sequence reconstruction. The entire decoder uses two such residual blocks. A skip connection is also used between the encoder and the decoder. The feature maps obtained from each convolutional layer on the left in the U-Net network will be concatenated to the corresponding upsampling layer using skip connections. The use of skip connections can better integrate low-level features and high-level features to avoid information loss.

Finally, in order to further improve the accuracy of feature extraction, we added CBAM to the above-mentioned improved U-Net. We added CBAM between the encoder and the decoder. The feature sequence output by the encoder will be optimized by CBAM and then passed into the decoder as input for decoding.

We input the pituitary tumor image sequence into the encoder to generate the feature sequence and used CBAM to further optimize it. Then, we used the decoder to reconstruct the spatial sequence. Finally, we compared the generated image with the original image at the pixel level. The more similar the two are, the more representative the extracted feature sequence is and the more it shows that the model has learned the features of the pituitary tumor image sequence well. This is the entire feature extraction process, and the extracted feature sequence will be used for further classification.

#### 2.4.2. Multisequence Pituitary Tumor Classification Model

The pituitary tumor image feature sequence extracted by CBAM_U-Net is a low-dimensional data sequence, which is strictly arranged in the order of image slices. Therefore, we used CRNN-based classifiers for the final classification of pituitary tumor texture. CRNN is composed of CNN and RNN and can capture the information of adjacent slices, which is more suitable for sequence data. We input the feature map sequence extracted by the CBAM_U-Net-based feature extractor into the CRNN-based classifier to obtain the classification result of pituitary tumor texture.

The final multisequence pituitary tumor texture classification model is shown in Figure 4.

## 3. Results

### 3.1. Experiment Platform and Dataset

The experimental running environment is as follows: the operating system is Windows 10, the processor is 2.10 GHz Intel Xeon (dual core), the memory capacity is 64 GB, the development environment is PyCharm, the deep learning framework is Keras, the programming language is Python, and the 5graphics card is GeForce RTX 2080Ti (three cores).

The pituitary tumor image dataset used in our experiment was provided by the local affiliated hospital. Each patient contains two modalities: T1 and T2. There are a total of 374 patients, of which 137 have labels (90 soft texture, 47 hard texture). The labels of each patient's pituitary tumor image are divided into two levels: soft texture and hard texture.

### 3.2. CycleGAN-Based Multisequence Data Amplification

The image data of 374 patients used in this experiment included 280 T1 MRI spatial sequences and 94 T2 MRI spatial sequences. The T2 MRI spatial sequence was severely lost. We trained CycleGAN for 90 epochs using the complete data of the image sequence and used the trained CycleGAN model to augment the image data of pituitary tumors with incomplete T1 or T2 sequences. The domain converter converted the T1/T2 domain to the T2/T1 domain. Finally, we expanded the slices of each patient to 24 (12 T1 slices, 12 T2 slices).  Figure 5 shows the test results of the existing T1 and T2 image pairs.

The Figure 5 shows the existing pairs of original T1 and T2 images and their images converted by CycleGAN. We can see that the converted images are very similar to the original images in their corresponding domains.

### 3.3. Amplification of Pituitary Tumor Data Based on Texture Analysis and Pseudo-Label Learning

Among the 374 cases of pituitary tumor image data amplified by CycleGAN, only 137 cases had labels, and the rest were unlabeled. In order to expand experimental data and improve data utilization, we used the texture analysis+pseudo-label learning method to label the remaining 237 pituitary tumor data.

#### 3.3.1. Texture Analysis

In this experiment, FireVoxel software was used to extract regions of interest (ROI) for pituitary tumors, as shown in Figure 6.

According to the literature [10–12], the feature parameters extracted by FireVoxel software are mainly mean, standard deviation, inhomogeneity, skewness, kurtosis, and entropy. We performed independent *t*-tests for these parameters. When *P* < 0.05, it indicates that the parameters are statistically significant.

The experiment used SPSS 22.0 software for statistical analysis. Among them, kurtosis (T1), inhomogeneity (T2), and entropy (T2) are statistically significant. The ROC curves of these characteristics are shown in Figure 7.

The specific data is shown in Table 1:

It can be seen from the figures and table that the entropy value of the T2 mode is more effective for judging the soft and flexible texture of pituitary tumors. After analysis, there is a judgment value for entropy statistics, which is 3.91. When the entropy value of the pituitary tumor is less than 3.91, it is judged to be hard. When it is greater than 3.91, it is judged to be soft, and 237 cases of the pituitary tumor without labels were labeled with this criterion.

#### 3.3.2. Pseudo-Label Learning

After labeling the pituitary tumors analyzed by texture features, we used the pseudo-label learning method to further evaluate the labels of texture analysis and made the final labels to expand the dataset. The experiment used part of the data labeled by texture analysis and part of the data with real labels to synthesize a new training set to train the GRU model. The training process of the GRU model used in pseudo-label training is shown in Figures 8 and 9. When epoch reached 55, the model converged and reached the optimal.

We used the trained model to predict 237 cases of unlabeled data, and the prediction result is shown in Figure 10.

There are 200 cases of soft texture label and 37 cases of hard texture label. We integrated pseudo-labeled data with labeled data and finally got a total of 374 cases of pituitary tumor data, of which 290 cases are soft and 84 cases are hard.

### 3.4. Pituitary Tumor Texture Image Classification Based on Adaptively Optimized Feature Extraction

After data augmentation and pseudo-label labeling, this paper uses a feature extractor based on CBAM_U-Net to extract features from the preprocessed pituitary tumor image data and uses a CRNN-based classifier for texture classification. In order to ensure the effectiveness of the feature extractor, we trained the CBAM_U-Net model and the U-Net model 150 epochs for comparison. Networks were implemented using an adaptive moment estimation optimizer (Adam) and a mean square error loss function (MSE). The initial learning rate was set to 10^−5^ with a batch size of 4. The training process of the models is shown in Figure 11.

As can be seen from the figures, when the models were trained for 150 epochs, the accuracy of the CBAM_U-Net feature extraction model was higher than that of the U-Net feature extraction model, and the convergence speed of loss was faster and the minimum value was lower. It can be seen that adding CBAM makes the improved U-Net model more superior in unsupervised feature extraction.

We put three kinds of pituitary tumor image sequences (multisequence, T1, and T2) into CBAM_U-Net for feature extraction, then put the results into CRNN for training, and divided them into three models, namely, the multisequence model, the T1 domain model, and the T2 domain model. The CRNN classifier was implemented using an adaptive moment estimation optimizer (Adam) and a cross entropy loss function (CE). The batch size was set to 10. We compared them experimentally.

1. T1 domain model: only the MRI spatial sequence of the T1 domain was used in the experiment, including the MRI spatial sequence of the T1 domain generated by CycleGAN
2. T2 domain model: only the MRI spatial sequence of the T2 domain was used in the experiment, including the MRI spatial sequence of the T2 domain generated by CycleGAN
3. Multisequence model: MRI spatial sequences of T1 and T2 domains were used in the experiment, including the MRI spatial sequences of T1 and T2 domains generated by CycleGAN

Figures 12–14 show the training process of the T1 domain, T2 domain, and multisequence model, respectively.

As shown in the figures, we divided the pituitary tumor image data into a training set (80%) and a test set (20%). The test set was randomly selected from the labeled dataset and did not contain pseudo-labeled data. The experiment was repeated 4 times in the T1 domain, T2 domain, and multisequence domain. We recorded each classification accuracy and AUC (95% CI) to calculate the final average and variance. The detailed information is shown in Table 2.

Table 3 shows the classification accuracy and AUC (95% CI) before and after amplification of the pseudo-label data.

In addition, the experiment not only added CBAM between the encoder and the decoder but also added CBAM to different places such as the encoder or the skip connections to compare its different effects. The final results are shown in Table 4. As can be seen from the table, the effect was best when CBAM was added between the encoder and the decoder.

### 3.5. Compared with Other Models

With the application and development of deep learning, many excellent feature extraction models have emerged. The quality of tumor feature extraction has a great correlation with the final classification result. In order to further illustrate the effectiveness of the pituitary tumor classification method based on CBAM_U-Net, we reimplemented some commonly used classification models on brain tumor image data.  Table 5 shows the classification results of the classification model proposed in this paper and some commonly used classification models on brain tumor image data. All results are based on the same cross validation scheme and test set.

As can be seen from the table, the model combining the feature extractor based on CBAM_U-Net and the classifier based on CRNN has the highest classification accuracy. Improved encoders and decoders can help further mine the information of images. Skip connections can combine low-level and high-level features. CBAM can strengthen feature propagation, reduce redundant information that is not related to tumors, and focus on useful information. CRNN can capture the information of adjacent slices of sequence data. The combination of these techniques enables us to improve the classification model accuracy to a certain extent and reduce the amount of network calculations. In addition, the classification model in this paper is more suitable for small-size medical image datasets than those transformer-based models that often require a large amount of data. This comparative experiment shows the great potential and good application prospects of our proposed method in grading pituitary tumor texture.

## 4. Discussion

This study designed a series of experiments to classify brain tumor texture and took MRI of the pituitary tumor as an example. First, for incomplete sequence data, this study used CycleGAN to augment the imaging data of pituitary tumors lacking T1 or T2 sequences. CycleGAN converted T1/T2 sequences to T2/T1 sequences. This paper tested it on existing pairs of T1 and T2 images to verify the success of the method. The texture features extracted from the converted T1/T2 sequence are closer to the T2/T1 sequence. Secondly, we used the method of texture analysis+pseudo-label learning to label the unlabeled pituitary tumor image data. This method first uses texture analysis to initially label unlabeled data and then uses GRU-based pseudo-label learning to complete pseudo-label labeling. This method incorporates statistical features and machine-learned features to improve the reliability of pseudo-label labeling and the utilization of pituitary tumor data. This study used FireVoxel software to extract feature parameters in the texture analysis part of pseudo-label labeling. A total of 12 basic features were extracted from the T1 and T2 images, and the useful features after screening were used for initially labeling of unlabeled data. In future work, we will devote to extracting more texture features and selecting features that are more relevant to brain tumor texture for pseudo-labeling.

This paper proposes an unsupervised feature extractor based on improved U-Net to extract the features of the pituitary tumor image sequence. The feature extractor uses dense blocks and residual blocks to optimize feature extraction to extract more representative features. In the experiment, the pituitary tumor image sequence was input into the encoder of the feature extractor for feature extraction and then restored by the decoder. The generated image sequence was compared with the original input image sequence. The more similar the two, the better the extracted features. This paper also introduces CBAM to the feature extractor. The attention mechanism can help models pay attention to useful information and suppress useless information to improve the reliability and efficiency of model feature extraction. CBAM is an attention mechanism that pays attention to both the spatial and the channel. Compared with the attention mechanisms that only pay attention to a certain aspect, it has a better effect. In future work, we will also try and improve more attention mechanisms to improve the classification model proposed in this paper. Finally, we input the extracted pituitary tumor features into the CRNN-based classifier for the final pituitary tumor texture classification. The entire classification model is end-to-end without the need for tumor presegmentation. In addition, this method is based on image sequences rather than 2D (slice) methods. We repeated the experiment 4 times and tested it on the labeled test set to obtain the classification accuracy and AUC (95% CI). Experimental results and comparative experiments show that our method has advantages in the classification of pituitary tumor texture. This method can also be applied to other types of brain tumors, such as glioma.

For larger-scale multisequence MRI data or multicenter study, the pseudo-label labeling method based on texture analysis and feature extractor proposed in this paper will also be applicable and can be used to provide direct input to other classification schemes. In conclusion, the method proposed in this paper can be applied to real clinical research to assist doctors in diagnosis and improve the efficiency of doctors' diagnosis. However, the imaging equipment used in different countries and regions is different, so there are still some differences in imaging and subsequent texture analysis. In addition, due to the privacy of medical images, it is difficult to collect a variety of large datasets. Therefore, designing a more versatile model is still a future research direction.

## 5. Conclusion

This paper proposes a brain tumor texture classification method based on pseudo-label learning and optimized feature extraction and takes pituitary tumors as an example. The experiment finally achieved 94.23% of average accuracy and 0.976 of average AUC (95% CI). Comparative experiments show that compared to some existing methods, our proposed method has more advantages and can improve the classification efficiency while improving the classification accuracy. This study shows great potential and good application prospects of our method in helping clinical diagnosis of brain tumors.

## Figures and Tables

**Figure 1:** Generator architecture.

**Figure 2:** Discriminator architecture.

**Figure 3:** Pseudo-label learning.

**Figure 4:** Multisequence pituitary tumor classification model.

**Figure 5:** Visualization of training results.

**Figure 6:** ROI.

**Figure 7:** Texture feature ROC.

**Figure 8:** Training accuracy of the pseudo-label model.

**Figure 9:** Training loss of the pseudo-label model.

**Figure 10:** Pituitary tumor data distribution.

**Figure 11:** Multisequence feature extraction model.

**Figure 12:** T1 domain image classification model training.

**Figure 13:** T2 domain image classification model training.

**Figure 14:** Multisequence image classification model training.

**Table 1:** Characteristic value statistics of pituitary tumors.

	AUC	*P* (<0.05)
Inhomogeneity (T2)	0.732	0.020
Entropy (T2)	0.828	0.010
Kurtosis (T1)	0.713	0.023

**Table 2:** Pituitary tumor classification accuracy.

	Multisequence	T1 domain	T2 domain
Accuracy (%)	94.23 ± 1.19	90.33 ± 1.28	89.00 ± 1.68
AUC (95% CI)	0.976 ± 1.44	0.918 ± 3.60	0.877 ± 3.75

**Table 3:** Comparison of accuracy before and after amplification of pseudo-label data.

	137 cases of data	374 cases of data
Accuracy (%)	91.08 ± 2.06	94.23 ± 1.19
AUC (95% CI)	0.930 ± 3.84	0.976 ± 1.44

**Table 4:** Comparison of accuracy of CBAM in different positions.

	Between the encoder and decoder	Encoder	Skip connections	Without CBAM
Accuracy (%)	94.23 ± 1.19	90.67 ± 1.89	89.33 ± 2.18	89.00 ± 2.00
AUC (95% CI)	0.976 ± 1.44	0.949 ± 1.07	0.953 ± 1.76	0.913 ± 2.77

**Table 5:** Comparisons of classification results of different methods.

Feature extraction	Texture classification	Accuracy (%)	Time (s)
—	VGG	71.89	119
—	ResNet	79.33	108
—	DenseNet	81.39	105
—	ViT	86.67	197
—	CRNN	77.33	72
Autoencoder (DenseNet+ResNet)	CRNN	87.34	46
U-Net (DenseNet+ResNet)	CRNN	89.00	46
U-Net (DenseNet+ResNet)+CBAM	CRNN	94.23	49

## Data Availability

The datasets generated during and analyzed during the current study are not publicly available due to hospital data confidentiality but are available from the corresponding author on reasonable request.
